The article "Healthcare's Sustainable Resource Planning Using Neutrosophic Goal Programming" was published in 2022. Journal: J Healthc Eng.

# Healthcare's Sustainable Resource Planning Using Neutrosophic Goal Programming

**DOI:** 10.1155/2022/3602792

**Published:** 2022-01-07

**Authors:** Ibrahim M. Hezam, Sarah A. H. Taher, Abdelaziz Foul, Adel Fahad Alrasheedi

**Affiliations:** Statistics & Operations Research Department, College of Sciences, King Saud University, Riyadh, Saudi Arabia

## Abstract

We develop neutrosophic goal programming models for sustainable resource planning in a healthcare organization. The neutrosophic approach can help examine the imprecise aspiration levels of resources. For deneutrosophication, the neutrosophic value is transformed into three intervals based on the truth, falsity, and indeterminacy-membership functions. Then, a crisp value is derived. Moreover, multi-choice goal programming is also used to get a crisp value. The proposed models seek to draw a strategic plan and long-term vision for a healthcare organization. Accordingly, the specific aims of the proposed flexible models are meant to evaluate hospital service performance and to establish an optimal plan to meet the growing patient needs. As a result, sustainability's economic and social goals will be achieved so that the total cost would be optimized, patients' waiting time would be reduced, high-quality services would be offered, and appropriate medical drugs would be provided. The simplicity and feasibility of the proposed models are validated using real data collected from the Al-Amal Center for Oncology, Aden, Yemen. The results obtained indicate the robustness of the proposed models, which would be valuable for planners who could guide healthcare staff in providing the necessary resources for optimal annual planning.

## 1. Introduction

Optimizing existing resources in health organizations is critical to meeting the needs of patients. At the same time, organizations must develop a future strategic plan of the existing resources commensurate with the predicted growth in the number of patients. Optimization approaches can support planning and decision-making at all levels. One of these approaches is goal programming in resources planning. Goal programming is a multi-objective optimization tool that helps a solution to move toward an ideal goal. In recent years, the use of goal programming has become more widespread, especially for analyzing and evaluating healthcare organizations. Numerous authors have considered goal programming to optimize the resources in health organizations. Parra et al. (1997) [1] proposed a goal programming model to evaluate the performance of a surgical service at a local general hospital. The authors aimed to improve the service under the available resources—for example, spatial occupation, staff availability, and financial support. Munoz et al. (2018) [2] improved a mathematical model based on goal programming to evaluate proposals in order to help in the selection of a mix of proposals. The main function of goal programming is the incorporation of strategic goals that support the vision and objectives of institutes. The model is applied using real data obtained from the Clinical and Translational Science Institute (CTSI) at Pennsylvania State University. Blake and Carter (2002) [3] proposed two linear goal programming models. The first model is used to determine case mix and volume for physicians under fixed service costs conditions. The second model addresses case-mix decisions as a commensurate set of practice changes for physicians. The trade-offs between case-mix and case costs are balanced using the proposed models and minimizing disturbance in order to preserve physician income. Rifai and Pecenka (1990) [4] applied goal programming to allocate resources in healthcare planning. Minimizing idle capacity and maximizing the profit are the main goals in this work. Kwak and Lee (2002) [5] proposed a multi-criteria mathematical programming model to evaluate strategic planning in a business process. This model is also based on goal programming. The goal levels are identified and prioritized using the analytic hierarchy process. Similarly, Lee and Kwak (1999) [6] presented a goal programming model for designing and evaluating effective information resource planning in a healthcare system. The proposed model addressed the multiple conflicting goals of a healthcare system and the multi-dimensional aspects of resource allocation planning. Also, the model allows flexibility of decision-making in resource allocation. The goals are decomposed and prioritized with respect to the corresponding criteria using the analytic hierarchy process. Grigoroudis and Phillis (2013) [7] proposed a nonlinear programming model to improve the health level of a population under several constraints. The system of systems approach is used to model the hierarchical structure of healthcare systems as well as for dynamic budget allocation for a national healthcare system in order to develop optimal policies. Lee and Kwak (2011) [8] developed a multi-criteria decision-making model for strategic enterprise resource planning adoption by considering both financial and nonfinancial business factors. Turgay and Taşkın (2015) [9] developed a fuzzy mixed goal programming model to optimize the healthcare organization's resource allocation problem in an uncertain environment.

The article "Healthcare's Sustainable Resource Planning Using Neutrosophic Goal Programming" was published in 2022. Journal: J Healthc Eng.

The use of neutrosophic concept theory in goal programming was first introduced by Hezam et al. (2016) [10]. For more information on the works related to neutrosophic goal programming, see Munoz et al. (2018), Islam and Kundu (2018), Maiti et al. (2019), Sarma et al. (2019), Dey and Roy (2017), Pramanik and Banerjee (2018), and Al-Quran and Hassan (2017) [2, 11–17].

At the same time, in conflict zones and poor communities, health organizations face difficulty meeting the population's needs [18]. There is an urgent need to provide excellent and comprehensive high-quality service for all patients under limited resources. In this regard, cancer is one of the most common diseases globally. Its treatment requires specialized experts, medical drugs, as well as exorbitant costs and time. In recent years, the number of people needing oncology services has increased significantly, especially in Yemen. Particularly, the country's growing population is facing health threats from the hazardous habit of chewing khat as well as pesticides used for growing the khat plant. The lack of health education, as well as early detection of tumors, also exacerbates the issue. Moreover, Yemen is a poor country that is suffering from ongoing conflicts. It has a dearth of human, material, and financial resources. Hence, the number of specialized oncology centers in Yemen is limited and, thus, does not meet the needs of oncology patients. As a result, most patients travel abroad for treatment. The Al-Amal Center for Oncology is one such specialized center for the treatment of tumors in Yemen. A large number of patients are treated by these health centers, which have limited resources. These complexities are reflected in the health facilities, making our data inaccurate, lacking, or ambiguous. Hence, we use the neutrosophic concept in this study.

In this article, we propose neutrosophic goal programming models for evaluating and optimizing the existing resources of health organizations and for optimal future planning. The main strategic goals to design the proposed models are (a) optimizing the center's resources; (b) matching the center service with the requirements of patients by providing high-quality services and appropriate medical drugs as well as reducing the waiting time; and (c) planning to meet the ideal center requirements by increasing the center capacity according to the predicted growth of patients. The real data are obtained from the Al-Amal Center for Oncology, Aden, Yemen. We use the data to validate the proposed models.

The remaining paper is organized as follows.  Section 2 provides an overview of goal programming, dynamic goal programming, and multi-choice goal programming. Besides, it presents neutrosophic concepts and deneutrosophication. In Section 3, we formulate the proposed models, while a case study is presented in Section 4.  Section 5 reports the results and discussion, and then Section 6 concludes the study.

The article "Healthcare's Sustainable Resource Planning Using Neutrosophic Goal Programming" was published in 2022. Journal: J Healthc Eng.

## 2. Theory

### 2.1. Goal Programming

Goal Programming is the most known method in multiple-criteria decision-making, proposed by Charnes and Cooper (1961). Goal programming is a generalization of linear programming that handles multiple conflicting objective measures, where a target is set for each measure to be achieved. The new objective function, or the “achievement function,” seeks to minimize unwanted deviations from aspiration levels or a set of target values.

We can introduce two types of constraints in goal programming: hard and soft constraints. Hard constraints are the system constraints that cannot be violated (e.g., system resources and relational model constraints). In contrast, soft constraints are associated with prespecified targets. Both negative and positive deviational variables are added to these constraints and the undesired deviations are included in the objective function to be minimized.

The priority of goal programming is to satisfy the hard constraints before soft constraints. The preference structures to minimize the undesired deviations require different methods: preemptive, nonpreemptive, and Tchebycheff. The preemptive variant is used when there is a natural priority structure to the decision-maker(s) preferences, the nonpreemptive variant is used when each unwanted deviation has a relative weight (which can be equal), and Tchebycheff goal programming is used when the maximum deviation from the target is minimized.

Consider the following model:

(1) $$\begin{array}{c} z=\min\sum_{l=1}^{L}w_{l}\left(n_{l}+p_{l}\right), \end{array}$$

(2) $$\begin{array}{c} f_{l}\left(x\right)+n_{l}-p_{l}=g_{l},\;\forall l\in L, \end{array}$$

(3) $$\begin{array}{c} n_{l}\times \;p_{l}=0,\;\forall l\in L, \end{array}$$

(4) $$\begin{array}{c} Ax\leq b, \end{array}$$

(5) $$\begin{array}{c} x\geq 0,\;\;n_{l}, \end{array}$$

where *g*_*l*_ is specific goal of the objective function *f*_*l*_(*x*)∀*l* ∈ *L*.*w*_*l*_ is the penalty weight. *n*_*l*_  and  *p*_*l*_ are the under- and upper achievements of the *l*^th^ goal, respectively. Equation (1) represents the objective function that minimizes the sum of the positive/negative deviations for each goal. Equation (2) is related to the decision-maker's goals and computes the respective positive and negative deviations from each goal. Equation (3) ensures that at least one of the deviations must be equal to zero. Equation (4) relates to the system constraints in the decision space. Equation (5) ensures that all decision variables are nonnegative.

The article "Healthcare's Sustainable Resource Planning Using Neutrosophic Goal Programming" was published in 2022. Journal: J Healthc Eng.

### 2.2. Dynamic Goal Programming

Dynamic goal programming allows for a target value to be dynamic. This approach is used to evaluate along a planning period. References [19–21] addressed the dynamic goal programming where the target values are changed as per the planning period:

(6) $$\begin{array}{c} z=\min\sum_{l=1}^{L}\sum_{t=1}^{T}w_{t}\left(n_{lp}+p_{lp}\right),\\ f_{l}\left(x\right)+n_{lt}-p_{lt}=g_{lt},\;\forall l\in L,\;\forall t\in T,\\ n_{lt}\times \;p_{lt}=0,\;\forall l\in L,\;\forall t\in T,\\ Ax\leq b,\\ x\geq 0,n_{lt},\;p_{lt}\geq 0,\;\forall l\in L,\;\forall t\in T, \end{array}$$

where *g*_*lt*_ is specific goal of the objective function *f*_*l*_(*x*)∀*l* ∈ *L* per period *t*.

### 2.3. Multi-Choice Goal Programming

Multi-choice goal programming was proposed by Chang (2007) [22]. In this case, decision-makers are allowed to define multi-choice aspiration levels for each target. The decision-maker can use the multi-choice model as a decision aid to make better decisions for a given problem. The mathematical model is as follows:

(7) $$\begin{array}{c} \min\sum_{l=1}^{L}\left|f_{l}\left(x\right)-g_{l1}\text{ or }g_{l2}\text{or }\ldots \text{ or }g_{lm}\right|. \end{array}$$

Subject to

(8) $$\begin{array}{c} X\in F\left(F\text{ is a feasible set}\right). \end{array}$$

Here, there are multi aspiration levels (*g*_*l*1_ or *g*_*l*2_or  … or *g*_*lm*_). This model can be reformulated as:

(9) $$\begin{array}{c} \min n_{l}+p_{l},\\ f_{l}\left(x\right)+n_{l}-p_{l}=\sum_{j=1}^{m}b_{lj}S_{lj}\left(B\right),\;\forall l\in L,\\ S_{lj}\left(B\right)\in R_{l}\left(x\right),\;\forall l\in L,\\ n_{lt}\times \;p_{lt}=0,\;\forall l\in L,\;\forall t\in T,\\ Ax\leq b,\\ x\geq 0,n_{lt},\;p_{lt}\geq 0,\;\forall l\in L,\;\forall t\in T, \end{array}$$

where *b*_*lj*_ is the *j*th aspiration level of the *l*th goal and *S*_*lj*_(*B*) indicates the function of the binary serial number; *R*_*l*_(*x*) is the function of resources boundaries. For three aspiration levels, the first constraint of model (9) can be reformulated as the following constraints:

(10) $$\begin{array}{c} f_{l}\left(x\right)+n_{l}-p_{l}=g_{l1}b_{1}b_{2}+g_{l2}b_{1}\left(1-b_{2}\right)+g_{l3}\left(1-b_{1}\right)b_{2},\\ b_{1}+b_{2}>0,\\ b_{1},b_{2}\in \left\{0,1\right\}. \end{array}$$

Constraint (10) makes at least *b*_1_  or  *b*_2_ not equal zero. Therefore, only three choices—*g*_*l*1_,  *g*_*l*2_, or  *g*_*l*3_— are yielded.

### 2.4. Neutrosophic Concept

In real applications, the uncertainty of the parameters is common in mathematical computations. Uncertainty arises owing to imprecise and inconsistent data. Zadeh proposed the fuzzy theory in 1965 to deal with these kinds of data [23]. However, fuzzy sets consider only the truth-membership function that is unable to efficiently represent accurate information. A new membership function, called falsity-membership function, was later developed by Atanassov (1986) [24], who introduced the intuitionistic fuzzy set. Nevertheless, this technique too was limited by drawbacks in decision-making. In 1998, Smarandache [25] introduced a new concept named “neutrosophic” that considers three memberships functions: truth, indeterminacy, and falsity.

The article "Healthcare's Sustainable Resource Planning Using Neutrosophic Goal Programming" was published in 2022. Journal: J Healthc Eng.

#### 2.4.1. Neutrosophic Set

**Definition 1 .**

Let *X* ≠ ∅ be a universe set. A neutrosophic set *A* in  *X* is characterized by a truth-membership function $\mu_{{\tilde{A}}^{N}}$, an indeterminacy-membership function $\sigma_{A^{\tilde{N}}}$, and a falsity-membership function $\nu_{A^{\tilde{N}}}$:

(11) $$\begin{array}{c} {\tilde{A}}^{N}=\left\{x,\mu_{{\tilde{A}}^{N}}\left(x\right),\sigma_{{\tilde{A}}^{N}}\left(x\right),\upsilon_{{\tilde{A}}^{N}}\left(x\right);\;x\in X\right\}, \end{array}$$

where $\mu_{{\tilde{A}}^{N}}:X⟶]0^{-},\;1^{+}[$, $\sigma_{{\tilde{A}}^{N}}:X⟶]0^{-},\;1^{+}[$, and $\upsilon_{{\tilde{A}}^{N}}:X⟶]0^{-},\;1^{+}[$ represent the degrees of the truth-, indeterminacy-, and falsity-membership functions, respectively. No restriction exists on the sum of $\mu_{{\tilde{A}}^{N}}$, $\;\sigma_{{\tilde{A}}^{N}}$, and $\;\nu_{{\tilde{A}}^{N}}$. Thus, $0^{-}\leq \mu_{{\tilde{A}}^{N}}\left(x\right)+\;\sigma_{{\tilde{A}}^{N}}\left(x\right)\;+\;\nu_{{\tilde{A}}^{N}}\left(x\right)\leq 3^{+}$ for *x* ∈ *X*

**Definition 2 .**

A set (*α*, *β*, *γ*) − *cuts*, generated by ${\tilde{A}}^{N}$, where *α*, *β*, *γ* ∈ [0,1] are a fixed number such that *α*+*β*+*γ* ≤ 3 is defined as:

(12) $$\begin{array}{c} {\tilde{A}}_{\alpha ,\beta ,\gamma }^{N}=\left\{\begin{array}{cc} \langle x,\mu_{{\tilde{A}}^{N}}\left(x\right),\sigma_{{\tilde{A}}^{N}}\left(x\right),\upsilon_{{\tilde{A}}^{N}}\left(x\right)\rangle ;\; & x\in X,\\ \mu_{{\tilde{A}}^{N}}\left(x\right)\geq \alpha ,\;\sigma_{{\tilde{A}}^{N}}\left(x\right)\leq \beta ,\;\upsilon_{{\tilde{A}}^{N}}\left(x\right)\leq \gamma ;\; & \alpha ,\beta ,\gamma \in \left[0,1\right], \end{array}\right. \end{array}$$

where (*α*, *β*, *γ*) − *cuts*, denoted by ${\tilde{A}}_{\alpha ,\beta ,\gamma }^{N}$, is defined as the crisp set of elements *x* that belong to ${\tilde{A}}^{N}$ at least to the degree *α* and that belongs to ${\tilde{A}}^{N}$ at most to the degree *β*  and  *γ*.

#### 2.4.2. Generalized Triangular Neutrosophic Number

A generalized triangular neutrosophic number (GTNN) ${\tilde{\tau }}_{a}^{N}=\left(a,\;l_{\mu },r_{\mu };w_{a}\right),\left(a,\;l_{\sigma },r_{\sigma };u_{a}\right),\left(a,\;l_{\nu },r_{\nu };y_{a}\right)$ is a special neutrosophic set on a real number set *ℜ* whose degree of truth, indeterminacy, and falsity are given by:

(13) $$\begin{array}{c} \mu_{{\tilde{\tau }}_{a}^{N}}\left(x\right)=\left\{\begin{array}{cc} \frac{x-a+l_{\mu }}{l_{\mu }} & \;a-l_{\mu }\leq x<a\\ w_{a} & x=a\\ \frac{a+r_{\mu }-x}{r_{\mu }} & \;a<x\leq a+r_{\mu }\\ 0 & \text{otherwise} \end{array}\right.,\\ \sigma_{{\tilde{\tau }}_{a}^{N}}\left(x\right)=\left\{\begin{array}{cc} \frac{\left(a-x\right)+u_{a}\left(x-a+l_{\sigma }\right)}{l_{\sigma }} & \;a-l_{\sigma }\leq x<a\\ u_{a} & x=a\\ \frac{\left(x-a\right)+u_{a}\left(a+r_{\sigma }-x\right)}{r_{\sigma }} & \;a<x\leq a+r_{\sigma }\\ 1 & \text{otherwise} \end{array},\right.\\ \nu_{{\tilde{\tau }}_{a}^{N}}\left(x\right)=\left\{\begin{array}{cc} \frac{\left(a-x\right)+y_{a}\left(x-a+l_{\nu }\right)}{l_{\nu }} & \;a-l_{\nu }\leq x<a\\ y_{a} & x=a\\ \frac{\left(x-a\right)+y_{a}\left(a+r_{\nu }-x\right)}{r_{\nu }} & \;a<x\leq a+r_{\nu }\\ 1 & \text{otherwise} \end{array},\right. \end{array}$$

where *l*_*μ*_,  *r*_*μ*_,  *l*_*σ*_, *r*_*σ*_,  *l*_*ν*_, and  *r*_*ν*_ are called the spreads of the truth-, indeterminacy-, and falsity-membership functions, respectively; and *a* is the mean value. *w*_*a*_ represents the maximum degree of the truth-membership function, while *u*_*a*_ and *y*_*a*_ represent the minimum degrees of the indeterminacy- and falsity-membership functions, respectively, such that they satisfy the conditions below:

(14) $$\begin{array}{c} 0\leq w_{a}\leq 1,\\ 0\leq u_{a}\leq 1,\\ 0\leq y_{a}\leq 1,\\ \;0\leq w_{a}+u_{a}+y_{a}\leq 3. \end{array}$$

The article "Healthcare's Sustainable Resource Planning Using Neutrosophic Goal Programming" was published in 2022. Journal: J Healthc Eng.

#### 2.4.3. (*α*, *β*, *γ*) − Cut Set of GTNN

**Definition 3 .**

An (*α*, *β*, *γ*) − *cut* set of GTNN ${\tilde{\tau }}_{a}^{N}=\left(a,\;l_{\mu },r_{\mu };w_{a}\right),\left(a,\;l_{\sigma },r_{\sigma };u_{a}\right),\left(a,\;l_{\nu },r_{\nu };y_{a}\right)$ is a crisp subset of *ℜ*, which is defined as:

(15) $$\begin{array}{c} {\left({\tilde{\tau }}^{N}\right)}_{a}^{\alpha ,\beta ,\gamma }=\left\{x:\mu_{{\left({\tilde{\tau }}^{N}\right)}_{a}}\left(x\right)\geq \alpha ,\sigma_{{\left({\tilde{\tau }}^{N}\right)}_{a}}\left(x\right)\leq \beta ,\upsilon_{{\left({\tilde{\tau }}^{N}\right)}_{a}}\left(x\right)\leq \gamma \right\}, \end{array}$$

where 0 ≤ *w*_*a*_ ≤ 1,0 ≤ *u*_*a*_ ≤ 1,0 ≤ *y*_*a*_ ≤ 1, and 0 ≤ *w*_*a*_+*u*_*a*_+*y*_*a*_ ≤ 3.

An *α* − cut  set of a GTNN ${\tilde{\tau }}_{a}^{N}$ is a crisp subset of *ℜ*, which is defined as:

(16) $$\begin{array}{c} {\left({\tilde{\tau }}^{N}\right)}_{a}^{\alpha }=\left\{x:\mu_{{\left({\tilde{\tau }}^{N}\right)}_{a}}\left(x\right)\geq \alpha \right\}, \end{array}$$

where 0 ≤ *α* ≤ *w*_*a*_.

The article "Healthcare's Sustainable Resource Planning Using Neutrosophic Goal Programming" was published in 2022. Journal: J Healthc Eng.

According to the definition of GTNN, it can be easily shown that ${\left({\tilde{\tau }}^{N}\right)}_{a}^{\alpha }=\left\{x:\mu_{{\left({\tilde{\tau }}^{N}\right)}_{a}}\left(x\right)\geq \alpha ,\right\}$ is a closed interval, defined by ${\left({\tilde{\tau }}^{N}\right)}_{a}^{\alpha }=\left[a_{L}\left(\alpha \right),a_{R}\left(\alpha \right)\right]$ where *a*_*L*_(*α*)=(*a* − *l*_*μ*_*a*__)+(*αl*_*μ*_*a*__/*w*_*a*_) and *a*_*R*_(*α*)=(*a*+*r*_*μ*_*a*__) − (*αr*_*μ*_*a*__/*w*_*a*_). The mean of ${\left({\tilde{\tau }}^{N}\right)}_{a}^{\alpha }$ is

(17) $$\begin{array}{c} a_{\text{mid}}\left(\alpha \right)=a+\frac{r_{\mu_{a}}-l_{\mu_{a}}}{2}\left[1-\frac{\alpha }{w_{a}}\right]. \end{array}$$

Similarly, a *β* and *γ* − cut  set of GTNN ${\tilde{\tau }}_{a}^{N}$ is a crisp subset of *ℜ*, which is defined as

(18) $$\begin{array}{c} {\left({\tilde{\tau }}^{N}\right)}_{a}^{\beta }=\left\{x:\sigma_{{\left({\tilde{\tau }}^{N}\right)}_{a}}\left(x\right)\leq \beta \right\},\\ {\left({\tilde{\tau }}^{N}\right)}_{a}^{\gamma }=\left\{x:\upsilon_{{\left({\tilde{\tau }}^{N}\right)}_{a}}\left(x\right)\leq \gamma \;\right\}. \end{array}$$

where *u*_*a*_ ≤ *β* ≤ 1, *y*_*a*_ ≤ *γ* ≤ 1

It follows from the definition that ${\left({\tilde{\tau }}^{N}\right)}_{a}^{\beta }$ and ${\left({\tilde{\tau }}^{N}\right)}_{a}^{\gamma }$ are closed intervals, denoted by ${\left({\tilde{\tau }}^{N}\right)}_{a}^{\beta }=\left[a_{L}\left(\beta \right),a_{R}\left(\beta \right)\right]$ and ${\left({\tilde{\tau }}^{N}\right)}_{a}^{\gamma }=\left[a_{L}\left(\gamma \right),a_{R}\left(\gamma \right)\right]$, which can be calculated as:

 
*a*_*L*_(*β*)=(*a* − *l*_*σ*_*a*__)+((1 − *β*)*l*_*σ*_*a*__/1 − *u*_*a*_) and *a*_*R*_(*β*)=(*a*+*r*_*σ*_*a*__) − ((1 − *β*)*r*_*σ*_*a*__/1 − *u*_*a*_)
 
*a*_*L*_(*γ*)=(*a* − *l*_*ν*_*a*__)+((1 − *γ*)*l*_*ν*_*a*__/1 − *y*_*a*_) and *a*_*R*_(*γ*)=(*a*+*r*_*ν*_*a*__) − ((1 − *γ*)*r*_*ν*_*a*__/1 − *y*_*a*_)

Thus, the means of ${\left({\tilde{\tau }}^{N}\right)}_{a}^{\beta }\text{ and }{\left({\tilde{\tau }}^{N}\right)}_{a}^{\gamma }$ are:

(19) $$\begin{array}{c} a_{\text{mid}}\left(\beta \right)=a+\frac{r_{\sigma_{a}}-l_{\sigma_{a}}}{2}\left[\frac{\beta -u_{a}}{1-u_{a}}\right], \end{array}$$

(20) $$\begin{array}{c} a_{\text{mid}}\left(\gamma \right)=a+\frac{r_{\nu_{a}}-l_{\nu_{a}}}{2}\left[\frac{\gamma -y_{a}}{1-y_{a}}\right]. \end{array}$$

#### 2.4.4. De-Neutrosophication

In this work, the neutrosophic parameters will be treatment using two methods. In the first method, the crisp value will be the average of the mean of the three intervals obtained from the (*α*, *β*, *γ*) − cut set of GTNN. The crisp value can be calculated as equation (21).

(21) $$\begin{array}{c} {\left(\tau^{N}\right)}_{a}^{\alpha ,\beta ,\gamma }=\frac{1}{3}\left(a_{\text{mid}}\left(\alpha \right)+a_{\text{mid}}\left(\beta \right)+a_{\text{mid}}\left(\gamma \right)\right),\\ =a+\frac{r_{\mu_{a}}-l_{\mu_{a}}}{6}\left[1-\frac{\alpha }{w_{a}}\right],+\frac{r_{\sigma_{a}}-l_{\sigma_{a}}}{6}\left[\frac{\beta -u_{a}}{1-u_{a}}\right],+\frac{r_{\nu_{a}}-l_{\nu_{a}}}{6}\left[\frac{\gamma -y_{a}}{1-y_{a}}\right]. \end{array}$$

It can be easily proven that for ${\tilde{\tau }}_{a}^{N}=\left(a,\;l_{\mu },r_{\mu };w_{a}\right),\left(a,\;l_{\sigma },r_{\sigma };u_{a}\right),\left(a,\;l_{\nu },r_{\nu };y_{a}\right)\in \text{GTNN}\left(ℜ\right)$ and for any *α* ∈ [0, *w*_*a*_], *β* ∈ [*u*_*a*_, 1], *γ* ∈ [*y*_*a*_, 1], where 0 ≤ *α*+*β*+*γ* ≤ 3:

(22) $$\begin{array}{c} {\left({\tilde{\tau }}^{N}\right)}_{a}^{\alpha ,\beta ,\gamma }={\left({\tilde{\tau }}^{N}\right)}_{a}^{\alpha }\wedge {\left({\tilde{\tau }}^{N}\right)}_{a}^{\beta }\wedge {\left({\tilde{\tau }}^{N}\right)}_{a}^{\gamma }, \end{array}$$

where the symbol ∧ denotes the minimum among ${\left({\tilde{\tau }}^{N}\right)}_{a}^{\alpha },{\left({\tilde{\tau }}^{N}\right)}_{a}^{\beta }\text{ and }{\left({\tilde{\tau }}^{N}\right)}_{a}^{\gamma }$

Figure 1 illustrates the membership functions for a generalized triangular neutrosophic number (NN).

The article "Healthcare's Sustainable Resource Planning Using Neutrosophic Goal Programming" was published in 2022. Journal: J Healthc Eng.

In the second method of the deneutrosophication, we employ multi-choice goal programming to select a crisp value in the three obtained intervals that led to the truth-, indeterminacy-, and falsity-membership functions [*a*_*L*_(*α*), *a*_*R*_(*α*)], [*a*_*L*_(*β*), *a*_*R*_(*β*)], and [*a*_*L*_(*γ*), *a*_*R*_(*γ*)], respectively. Thus, the multi-choice model will be employed to select one value from the three mean values that have been obtained using equations (17), (19) and (20).

## 3. Proposed Models

In this section, we formulate three goal programming models. First, we construct the basic goal programming model. We extend this model to include the neutrosophic concepts, whose parameters will be treated using the two methods in Section 2.4.4.

The nomenclature of the parameters and the variables we use herein are defined below:

Nomenclature

  Sets:
 
*n*={1,2,…, *n*}: Set of all the staff kinds, indexed by *i*;
 
*m*={1,2,…, *m*}: Set of all the medical device types, indexed by *j*;
 
*K*={1,2,…, *K*}: Set of all the medical drug types, indexed by *k*.
  Decision variables
 
*x*_*i*_: The number of *i* staff;
 
*y*_*j*_: The number of *j* medical devices;
 
*z*_*k*_: The number of *k* medical drugs;
 
*p*, *n*: The positive and the negative deviational variables;
 
*px*_*i*_, *py*_*j*_, *pz*_*k*_: The positive deviational variables associated with the corresponding variable *i*, *j*, *k*;
 
*nx*_*i*_, *ny*_*j*_, *nz*_*k*_: The negative deviational variables associated with the corresponding variable *i*, *j*, *k*;
 
*δ*_*j*_ ∈ {0,1}: A binary variable, where $\delta_{j}=\left\{\begin{array}{c} 1\text{ if }y_{j}>{\left(\text{TNE}\right)}_{j}\\ 0\text{ if }y_{j}\leq {\left(\text{TNE}\right)}_{j} \end{array}\right.\;\forall j$
 
*b*_*r*_: A binary variable ∀*r*;
 
*M*: A large number.
  Parameters
 
*c*_*i*_: The cost of *i* staff;
 
*cm*_*j*_: The cost of *j* medical devices;
 
*cd*_*k*_: The cost of *k* medical drugs;
 
*W*_*l*_: The weights of priority;
 
TB: The total budget;
 
TBS: The total budget for staff resources;
 
TBM: The total budget of the medical device resources;
 
TBD: The target budget of the medical drugs;
 
(TNS)_i_: The target number of *i* staff;
 
(TNM)_j_: The target number of the *j* medical devices;
 
(QD)_k_: The quantity demand of the *k* medical drugs;
 
SH: The number of shifts;
 
*t*: The number of years;
 
XP_day_: The estimated number of the patients per day;
 
(XR)_i_: The optimal ratio between the number of  *i* stuff and the patients;
 
(YR)_j_: The optimal ratio between the number of *j* medical device and the patients;
 
GR: The estimated growth rate of patients.

The article "Healthcare's Sustainable Resource Planning Using Neutrosophic Goal Programming" was published in 2022. Journal: J Healthc Eng.

### 3.1. Goal Programming Model (GP)

The goal programming model can be formulated as follows:

(23) $$\begin{array}{c} \min\;z=\sum_{l=1}^{4}\left(p_{l}+n_{l}\right),+\sum_{i=1}^{n}\left(nx_{i}+px_{i}\right),K+\sum_{j=1}^{m}\left(ny_{j}+py_{j}\right),+\sum_{k=1}^{K}\left(nz_{k}+pz_{k}\right). \end{array}$$

Subject to

(24) $$\begin{array}{c} \sum_{i=1}^{n}c_{i}x_{i}+\sum_{j=1}^{m}cm_{j}y_{j}+\sum_{k=1}^{K}cd_{k}z_{k}+n_{1}-p_{1}\leq \;TB, \end{array}$$

(25) $$\begin{array}{c} \sum_{i=1}^{n}c_{i}x_{i}+n_{2}-p_{2}\leq \mathrm{TBS}, \end{array}$$

(26) $$\begin{array}{c} \sum_{j=1}^{m}cm_{j}y_{j}+n_{3}-p_{3}\leq \;\mathrm{TBM}, \end{array}$$

(27) $$\begin{array}{c} \sum_{k=1}^{K}cd_{k}z_{k}+n_{4}-p_{4}\leq \mathrm{TBD}, \end{array}$$

(28) $$\begin{array}{c} z_{k}+nz_{k}-pz_{k}\geq {\left(\text{QD}\right)}_{k}\;\forall k, \end{array}$$

(29) $$\begin{array}{c} x_{i}+nx_{i}-px_{i}\geq {\left(\mathrm{TNS}\right)}_{i}, \end{array}$$

(30) $$\begin{array}{c} y_{j}+ny_{j}-py_{j}\geq {\left(\text{TNM}\right)}_{j},\;\forall j, \end{array}$$

(31) $$\begin{array}{c} y_{j}>{\left(\text{TNM}\right)}_{j}-\left(1-\delta_{j}\right)M, \end{array}$$

(32) $$\begin{array}{c} y_{j}<{\left(\text{TNM}\right)}_{j}+\delta_{j}M, \end{array}$$

(33) $$\begin{array}{c} \text{TBS}+cm_{j}-\left(1-\delta_{j}\right)M\leq \sum_{i=1}^{n}c_{i}x_{i}\leq TBS+cm_{j}+\left(1-\delta_{j}\right)M, \end{array}$$

(34) $$\begin{array}{c} \text{TBS}-\delta_{j}M\leq \sum_{i=1}^{n}c_{i}x_{i}\leq \text{TBS}+\delta_{j}M, \end{array}$$

(35) $$\begin{array}{c} x_{i},y_{j},z_{k}\in {\mathbb{Z}}^{+},\;\forall i,j,k. \end{array}$$

The objective function in equation (23) is to minimize unwished deviations from the targets. Unwished deviations in these models are the negative deviational variables. Positive deviations are also added to the objective function to avoid obtaining large, exaggerated deviations. This way, decision-makers can provide the obtained budgets. The constraint mentioned in equation (24) ensures that the total available budget is not exceeded. In the flexible model, the budget is dynamic, that is, it changes according to the annual growth rate of the number of patients. Thus, equation (36) is used to calculate the targeted total budget over *t* number of years.

(36) $$\begin{array}{c} \text{TB}=\text{ TB}+t\times \text{GR}\times \text{ TB.} \end{array}$$

As the number of patients increases with time, the total budget must be increased to cover all costs of the optimal staff, medical devices, and medical drugs that will optimally satisfy patients' demand. To achieve the maximum budget, that is, to attain the aspiration level total budget TB, the undesired variable *n*_1_ must be minimized. Constraints (25)–(27), respectively, guarantee the sub-budgets for the staff, medical devices, and medical drugs each, such that they are not violated.

The article "Healthcare's Sustainable Resource Planning Using Neutrosophic Goal Programming" was published in 2022. Journal: J Healthc Eng.

Similarly, in the flexible model, the sub-budgets change according to the growth of the number of patients. Thus, the dynamic sub-budgets of the staff, medical devices, and medical drugs change per year according to the following equations:

(37) $$\begin{array}{c} \text{TBS}=\text{TBS}+t\times \text{GR}\times \text{TBS},\\ \text{TBM}=\text{TBM}+t\times \text{GR}\times \text{TBM,}\\ \text{TBD}=\text{TBD}+t\times \text{GR}\times \text{TBD.} \end{array}$$

Constraint (28) allows for increasing the amount of the *k* medical drug coinciding with the number of patients annually. In the same way, the amount of the *k* medical drug will change with time based on the following dynamic equation:

(38) $$\begin{array}{c} {\left(\text{QD}\right)}_{k}={\left(\text{QD}\right)}_{k}+t\times \text{GR}\times {\left(\text{QD}\right)}_{k}. \end{array}$$

Constraints (29) and (30) relate to the optimal ratio between the number of patients to the number of staff and medical devices. For example, the optimal ratio between the number of patients to number of oncologists for optimal care is about 1 : 15. On the other hand, the number of patients can be predicted from the previous data using the prediction techniques. Thus, we can estimate the number of patients daily. Therefore, the number of oncologists should be not less than

(39) $$\begin{array}{c} x_{1}\geq {\left(\text{TNS}\right)}_{1}=\frac{\text{SH}}{{\left(\text{XR}\right)}_{1}}{\text{XP}}_{\text{day}}. \end{array}$$

Similarly, for all other staff and medical advices that must be not less than the required number according to constraints (29) and (30), the target number of staff and medical devices can be calculated by the following equations:

(40) $$\begin{array}{c} {\left(\text{TNS}\right)}_{i}=\frac{\text{SH}}{{\left(\text{XR}\right)}_{i}}{\text{XP}}_{\text{day}},\forall i,\\ {\left(\text{TNM}\right)}_{j}=\frac{\text{SH}}{{\left(\text{YR}\right)}_{j}}{\text{XP}}_{\text{day}},\;\forall j\;. \end{array}$$

We assume the importance of the availability of staff in the healthcare system and that medical devices have long-term durability. Therefore, constraints (31)–(34) transfers the surplus of the budget of the medical devices to the staff budget. This constraint investigates whether the medical device is available, and then shifts the budget of this type of device to the staff budget. Constraint (35) is related to the type of variables that must be integer variables.

The article "Healthcare's Sustainable Resource Planning Using Neutrosophic Goal Programming" was published in 2022. Journal: J Healthc Eng.

### 3.2. Neutrosophic Goal Programming Model (NGP)

The state of a country's economy can be expressed through its economic growth, stability, and stagnation. Thus, the total budget of any health center is affected by these economic states. Consequently, the sub-budgets will increase or decrease according to the economic state. Hence, the most suitable mathematical concept that expresses these states is the neutrosophic concept. In this subsection, we propose neutrosophic goal programming for healthcare planning. Three degrees are introduced in this case: acceptable, indeterminacy, and rejection.

The neutrosophic goal programming model is the extension of the goal programming model, where constraints (24)–(27) and (31)–(34) are rewritten as follows:

(41) $$\begin{array}{c} \sum_{i=1}^{n}c_{i}x_{i}+\sum_{j=1}^{m}cm_{j}y_{j}+\sum_{k=1}^{K}cd_{k}z_{k}+n_{1}-p_{1}\leq \;{\tilde{\text{TB}}}^{N},\\ \sum_{i=1}^{n}c_{i}x_{i}+n_{2}-p_{2}\leq {\tilde{\text{TBS}}}^{N},\\ \sum_{j=1}^{m}cm_{j}y_{j}+n_{3}-p_{3}\leq {\tilde{\text{TBM}}}^{N}\;,\\ \sum_{k=1}^{K}cd_{k}z_{k}+n_{4}-p_{4}\leq \;{\tilde{\text{TBD}}}^{N},\\ y_{j}>{\left(\text{TNM}\right)}_{j}-\left(1-\delta_{j}\right)M,\\ y_{j}<{\left(\text{TNM}\right)}_{j}+\delta_{j}M,\\ {\left(\tilde{\text{TBS}}\right)}^{N}+cm_{j}-\left(1-\delta_{j}\right)M\leq \sum_{i=1}^{n}c_{i}x_{i}\leq {\left(\tilde{\text{TBS}}\right)}^{N}+cm_{j}+\left(1-\delta_{j}\right)M,\\ {\left(\tilde{\text{TBS}}\right)}^{N}-\delta_{j}M\leq \overset{n}{\underset{i=1}{\sum }}c_{i}x_{i}\leq {\left(\tilde{\text{TBS}}\right)}^{N}+\delta_{j}M,\\ {\tilde{\text{TB}}}^{N}=\left(\text{TB},\;l_{\mu },r_{\mu };w_{\text{TB}}\right),\left(\text{TB},\;l_{\sigma },r_{\sigma };u_{\text{TB}}\right),\left(\text{TB},\;l_{\nu },r_{\nu };y_{\text{TB}}\right),\\ {\left(\tilde{\text{TBS}}\right)}^{N}=\left(\text{TBS},\;l_{\mu },r_{\mu };w_{\text{TBS}}\right),\left(\text{TBS},\;l_{\sigma },r_{\sigma };u_{\text{TBS}}\right),\left(\text{TBS},\;l_{\nu },r_{\nu };y_{\text{TBS}}\right),\\ {\left(\tilde{\text{TBM}}\right)}^{N}=\left(\text{TBM},\;l_{\mu },r_{\mu };w_{\text{TBM}}\right),\left(\text{TBM},\;l_{\sigma },r_{\sigma };u_{\text{TBM}}\right),\left(\text{TBM},\;l_{\nu },r_{\nu };y_{\text{TBM}}\right),\\ {\tilde{\text{TBD}}}^{N}=\left(\text{TBD},\;l_{\mu },r_{\mu };w_{\text{TBD}}\right),\left(\text{TBD},\;l_{\sigma },r_{\sigma };u_{\text{TBD}}\right),\left(\text{TBD},\;l_{\nu },r_{\nu };y_{\text{TBD}}\right), \end{array}$$

where ${\left(\tilde{A}\right)}^{N}$ denotes the neutrosophic number defined using constraint (41).

The article "Healthcare's Sustainable Resource Planning Using Neutrosophic Goal Programming" was published in 2022. Journal: J Healthc Eng.

### 3.3. Neutrosophic Multi-Choices Goal Programming Model (NMCGP)

In this model, we use multi-choice goal programming to deal with values obtained from the neutrosophic set. Hence, constraints (24)–(27) are rewritten as follows:

(42) $$\begin{array}{c} \sum_{i=1}^{n}c_{i}x_{i}+\sum_{j=1}^{m}cm_{j}y_{j}+\sum_{k=1}^{K}cd_{k}z_{k}+n_{1}-p_{1}\leq {\text{TB}}_{1}^{N}b_{1}b_{2}+{\text{TB}}_{2}^{N}b_{1}\left(1-b_{2}\right)+{\text{TB}}_{3}^{N}\left(1-b_{1}\right)b_{2},\\ \sum_{i=1}^{n}c_{i}x_{i}+n_{2}-p_{2}\leq {\text{TBS}}_{1}^{N}b_{3}b_{4}+{\text{TBS}}_{2}^{N}b_{3}\left(1-b_{4}\right)+{\text{TBS}}_{3}^{N}\left(1-b_{3}\right)b_{4},\\ \sum_{j=1}^{m}cm_{j}y_{j}+n_{3}-p_{3}\leq {\text{TBM}}_{1}^{N}b_{5}b_{6}+{\text{TBM}}_{2}^{N}b_{5}\left(1-b_{6}\right)+{\text{TBM}}_{3}^{N}\left(1-b_{5}\right)b_{6},\\ \sum_{k=1}^{K}cd_{k}z_{k}+n_{4}-p_{4}\leq \;{\text{TBD}}_{1}^{N}b_{7}b_{8}+{\text{TBD}}_{2}^{N}b_{7}\left(1-b_{8}\right)+{\text{TBD}}_{3}^{N}\left(1-b_{7}\right)b_{8},\\ b_{r}+b_{r+1}>0,\\ b_{r},b_{r+1}\in \left\{0,1\right\},\\ r\in \left\{1,2,,\ldots ,7\right\}, \end{array}$$

where  TB_1_^*N*^,  TB_2_^*N*^,  TB_3_^*N*^, TBS_1_^*N*^, TBS_2_^*N*^, TBS_3_^*N*^, TBM_1_^*N*^, TBM_2_^*N*^, TBM_3_^*N*^, TBD_1_^*N*^, TBD_2_^*N*^,  *an*  *d* TBD_3_^*N*^ can be obtained using equations (17), (19) and (20).

## 4. Case Study

For the case study, we collected and mined real data from the Al-Amal Center for Oncology in Aden, Yemen. Then, the number of patients was predicted daily, and the goals were set according to the predicted data.

The center was established in 2014 and covers an area of 50,000 km^2^. The center includes several departments and sections, such as outpatient clinics, inpatient section, laboratories and radiology department, early detection center, research center, intensive care, emergency section, a medical college, administrative, training, and staff housing.

The article "Healthcare's Sustainable Resource Planning Using Neutrosophic Goal Programming" was published in 2022. Journal: J Healthc Eng.

Al-Amal is one of the few specialized centers for oncology in Yemen. Owing to the increasing rates of cancer, this center faces immense challenges in providing the necessary supplies for staff, medical devices, and medical drugs.  Table 1 shows the increasing growth of the number of patients for the period between July 2015 and December 2017.

Based on the given data, the linear regression equation to predict the numbers of patients is XP=1227+3526*t*, where XP is the estimated number of patients and *t* is the number of years. Hence, the number of patients increases gradually with an average annual growth rate of 8%. That is, the estimated number of patients on a working day is XP_day_≅5+10*t*. Hence, the increasing number of patients daily under the existing budget requires more optimal use of resources. Moreover, we hope to increase the number of staffs, medical devices, and medical drugs as well, which would require increasing the budget. In the next step, increasing the total budget and sub-budgets would be a target, which would help meet the needs of growing patient numbers.

Table 2 shows the number of each kind of staff and the respective cost. The staff include oncologists, general doctors, radiologists, pharmacists, lab technicians, X-ray technicians, nurses, and other staff (other staff include remaining staff such as those in the administrative department).

Table 3 shows the number of each type of medical device and the respective cost. The medical devices include blood testing apparatus, chemistry apparatus, oncology indications, as well as ultrasonic, X-ray, mammogram, and other equipment (e.g., blood pressure- and blood sugar-testing devices as well as medical stethoscopes).  Table 4 shows the list of the medical drugs, including their name, size, price, type, quantities used, and doses.

The existing budget of the center for the staff, medical devices, and medical drug are US$135,600, US$45,260, and US$390,000, respectively, or US$570,860 in total.

## 5. Results and Discussion

In this section, we implement the three proposed models using LINGO 18.0 software. We use these models for planning the sustainable development of the Al-Amal center for Oncology, Aden, Yemen. The proposed models would help decision-makers to plan optimality, as it allows us to determine the optimal number of required staffs, devices, and medical drugs for every period. The optimal ratio between the number of patients to the number of staff/medical devices/quantity of the medical drugs are assumed and the proposed models are applied to eight periods, from 2018 to 2048.

The article "Healthcare's Sustainable Resource Planning Using Neutrosophic Goal Programming" was published in 2022. Journal: J Healthc Eng.

### 5.1. Results of the Goal Programming Model

The results of the first model are illustrated in Tables 5–10, where Table 5 shows the optimal budgets for each year and the ratio of each sub-budget of the total budget. Four budgets in this study are considered: total budget, staff budget, medical devices budget. and medical drugs budget. In the last column of this table, the growth rate for each budget is presented. The results indicate the need to increase the budget of the staff numbers, medical devices, and medical drugs by 13%, 6%, 9%, and 32%, respectively, annually.  Figure 2 illustrates the growth of the total budget as well as the other budgets.

Table 6 shows the optimal staff numbers that should be employed annually. Each row in this table indicates the years and the corresponding optimal staff number, each ratio of the total, and the corresponding cost for each. In the last row of this table, we observe an increase in the varying annual growth rates for each kind of staff, according to the corresponding optimal rate with respect to the number of patients. The growth rate for the total staff is 6%.

Figure 3 illustrates the optimal number of different staffs. Evidently, the number of nurses increases the most with time. Similarly, Tables 7 and 8 show the increasing number of medical devices and medical drugs, respectively.  Figure 4 illustrates the growth of the number of medical devices; we find that other equipment increases the most with time. The growth rate for the total number of medical devices is 4%, which is less than the total number of staff growth owing to converted constraints (31)–(34).

Table 9 shows the negative deviational variables. Almost all variables equal to zero except N1 and N4, which are equal to US$4,800. That is, in 2018, the optimal budget of the medical drugs must be decreased to US$385,200. All the remaining negative deviations are equal to zero and, hence, there is no need to record them in the table. In contrast, the nonzero positive deviational variables are reported in Table 10.

We find that the total budgets, staff, and medical devices should be increased further in order to provide high-quality service in expectation of the annual increase in patients. The positive deviations of medical drugs are equal to zero—its dynamic budget can sufficiently cover needs.

### 5.2. Results of the Neutrosophic Goal Programming Model

There are three states of an economy: growth, stability, and stagnation. The budgets are assumed in accordance with these states. That is, the budgets are increased in the optimism state; are left unchanged or changed only marginally in the stability state; and are decreased in the pessimism state. This allows us to represent the budgets using the neutrosophic concept.  Table 11 shows the values of the neutrosophic parameters. Then, equation (21) is used to give the deneutrosophic treatment to the obtained values.

The article "Healthcare's Sustainable Resource Planning Using Neutrosophic Goal Programming" was published in 2022. Journal: J Healthc Eng.

Table 12 shows the optimal different budgets for each year. The results indicate that the budgets' growth rate is 15% annually. There is a marginal increase in the growth rate in the goal programming model.  Table 13 shows that the optimal staff number should be determined yearly using this model. The growth rate for the total staff is 8%. There is a small decrease in the growth rate in the goal programming model. In the same way, Tables 14 and 15 show the increase in medical devices and medical drugs. We find that other equipment increases the most with time. The negative deviational variables are also equal to zero except N3, which is equal US$20,064 for 2018, as reported in Table 16. In contrast, the nonzero positive deviational variables are mentioned in Table 17.

### 5.3. Results of the Neutrosophic Multi-Choices Goal Programming Model

In this model, the multi-choice goal programming was applied to randomly select one value from the three values obtained from the neutrosophic membership functions.  Table 18 shows the three means for each budget obtained using equations (17), (19) and (20) with the same parameters reported in Table 11.

Tables 19–22 show the obtained values for all variables. Similarly, Figures 5–7 illustrate the growth in the budgets, staff, medical devices, and medical drugs. Notably, we observe the aliasing of the curves, in contrast to Figure 2, indicating the random selection of the values of binary variable *b* using multi-choice goal programming.

Overall, Table 23 summarizes the comparison between the three proposed models. The growth rates of the total budget and total staff numbers using the neutrosophic goal programming model were the highest, whereas the multi-choice model shows the highest growth rate of the number of medical devices. The growth rate of medical drugs for all proposed models is almost equal. The multi-choice model yields the least deviations. We now discuss the results obtained in 2048 as an example. The total budget, total staff, and total medical devices obtained using the multi-choice model are higher than those obtained using the other models. Similarly, in the same year, the multi-choice model yields the lowest summation of deviations. Figures 8–10 illustrate a comparison between the proposed models for staff growth, the increasing medical devices, and the increase in the demand for medicines for the period between 2018 and 2048, respectively.

The article "Healthcare's Sustainable Resource Planning Using Neutrosophic Goal Programming" was published in 2022. Journal: J Healthc Eng.

The case study shows that, in the three proposed models, the ratio of staff's budget to the total budget increases annually. In contrast, the ratio of the medical drugs' budget to the total budget decreases annually. Tables 5, 12, and 19 show that the ratios in 2018 are 28%, 34%, and 15% of the staff's budget from the total budget and 64%, 59%, and 76% of medical drugs' budget from the total budget, while the ratios in 2048 are 63%, 63%, and 63% of the staff's budget from the total budget and 26%, 25%, and 26% of medical drugs' budget from the total budget. The obtained results of the case study are almost similar. This convergence indicates the stability and robustness of the mathematical models.

On the other hand, the large numbers, in this case, have made significant differences unclear. In general, the results obtained using both neutrosophic goal programming models are more realistic and flexible than the results obtained without the neutrosophic approach. We thus introduced several scenarios for each period, allowing the decision-maker more flexibility to choose the most appropriate model that corresponds to other uncontrolled factors in this study. For example, the economy grew rapidly in a specific period, which would enable the decision-maker to choose the largest budget then; the converse holds true during periods of recession. Therefore, the proposed models in this study provide sustainable planning for several future periods.

## 6. Conclusions

In this paper, we proposed three models for solving healthcare planning problems. The proposed models were applied to a realistic case study of the Al-Amal Center for Oncology in Aden, Yemen. We used dynamic goal programming to predict the optimal solution for each variable in every period addressed in this article. Three models were eventually proposed: crisp, neutrosophic, and neutrosophic multi-choice goal programming. The goals addressed in the proposed models are related to the budget, the number of staffs and materials to perform the tasks efficiently. The proposed models yielded the optimum budget as well as the optimal number of staff and other medical supplies required to provide high-quality service for patients. Our results and insights thereof would be valuable for planners who could guide healthcare staff in providing the necessary resources for optimal annual planning. The diversity in the results obtained from the proposed models gives decision-makers the flexibility to make optimal decisions based on the state of the economy in each period. Although the proposed models were applied to healthcare planning, our approaches can be implemented on a large-scale healthcare system. Moreover, metaheuristics algorithms can be used to solve the models.

The article "Healthcare's Sustainable Resource Planning Using Neutrosophic Goal Programming" was published in 2022. Journal: J Healthc Eng.

## Figures and Tables

**Figure 1:** Graphical representation of membership functions for NN.

**Figure 2:** Budget growth using the GP model.

**Figure 3:** The staff growth using the GP model.

**Figure 4:** Medical devices growth using GP model.

**Figure 5:** Budget growth using the NMCGP model.

**Figure 6:** The staff growth using the NMCGP model.

**Figure 7:** The medical devices growth using the NMCGP model.

**Figure 8:** Comparison of staff growth between the proposed models.

**Figure 9:** Comparison of increase in devices between the proposed models.

**Figure 10:** Comparison of the growing demand for medicines between the proposed models.

**Table 1:** Number of patients (7/2015–12/2017).

Months	JAN.	FEB.	MAR.	APR.	MAY	JUN.	JUL.	AUG.	SEP.	OCT.	NOV.	DEC.	Total
2015	—	—	—	—	—	—	263	277	278	296	334	361	1809
2016	366	382	102	195	230	104	201	203	309	400	453	644	3589
2017	650	681	689	696	730	733	737	755	770	788	794	838	8861

**Table 2:** The number of staffs with corresponding costs.

Staff	*x*_1_	*x*_2_	*x*_3_	*x*_4_	*x*_5_	*x*_6_	*x*_7_	*x*_8_	Total
	Oncologists	General doctors	Radiologists	Pharmacists	Lab technician	X-ray technician	Nurses	Other staff	
Number of staffs	2	2	1	2	2	1	6	20	36
Cost ($)	9600	3840	5760	3360	3360	3120	2400	3600	
Total cost ($)	19200	7680	5760	6720	6720	3120	14400	72000	135600
(XR)_*i*_	15	20	10	100	10	30	4	10	

**Table 3:** The number of machines with corresponding costs.

Machines	*y*_1_	*y*_2_	*y*_3_	*y*_4_	*y*_5_	*y*_6_	*y*_7_	Total
	Blood Test	Chemistry apparatus	Oncology indications	Ultrasonic	X-ray	Mammogram	Other equipment	
Number of machines	1	1	1	1	1	1	200	206
Cost	4200	4800	6660	9600			100	
Total cost ($)	4200	4800	6660	9600			20000	45260
(YR)_*j*_	10	30	30	30	30	50	3	

**Table 4:** Medical drug data.

Medical drug names		The size of the medicine (cm^3^)	Drug Price ($)	Type of medication	Quantity 2016	Dose of medication
*z*_1_	Capecitabin	243	1.18	Tab	13503	500 mg
*z*_2_	Cisplatin -1-	128	1.67	Vial	80	10 mg
*z*_3_	Cisplatin -2-	212.5	6.04	Vial	484	50 mg
*z*_4_	Cyclophosphamide -1-	112	1.1	Vial	1061	500 mg
*z*_5_	Cyclophosphamide -2-	54	0.7	Vial	1049	200 mg
*z*_6_	Cyclophosphamide-3-	212.5	1.61	Vail	366	1000 mg
*z*_7_	Docitaxel -1-	150	9.69	Vial	610	20 mg
*z*_8_	Docitaxel -2-	282.6	18.98	Vial	694	80 mg
*z*_9_	Epirubicin -1-	37.5	4.66	Vial	155	10 mg
*z*_10_	Epirubicin -2-	112	18.7	Vial	605	50 mg
*z*_11_	Letrozole tabl.	178.5	0.25	Tab	4535	2.5 mg
*z*_12_	Paclitaxel -1-	128	31.45	Vial	210	150 mg
*z*_13_	Paclitaxel -2-	68.25	14.8	Vial	275	100 mg
*z*_14_	Paclitaxel -3-	54	6.66	Vial	155	30 mg
*z*_15_	Fluorouracil (5-fu)-1-	200	0.66	Vail	110	250 mg
*z*_16_	Fluorouracil (5-fu)-2-	262.5	1.38	Vail	226	500 mg
*z*_17_	Tamoxifen	95	0.12	Tab	6374	20 mg
*z*_18_	Thalidomide	80.325	1.35	Tab	778	100 mg
*z*_19_	Doxorubcin -1-	91.875	5.26	Vial	490	50 mg
*z*_20_	Doxorubcin -2-	58.5	1.66	Vial	756	10 mg
*z*_21_	Ifosphamid	211.75	4.85	Vial	152	1000 mg
*z*_22_	Zoledronic acid	58.5	15.82	Vial	213	4 mg
*z*_23_	Imatinib	44	1.4	Tab	2575	400 mg
*z*_24_	Biclutamide	33.8	0.82	Tab	2002	50 mg
*z*_25_	Carboplatin -1-	212.5	35.7	Vial	281	450 mg
*z*_26_	Carboplatin -2-	128	16.83	Vial	262	150 mg
*z*_27_	Gemcitabin -1-	128	29.06	Vial	411	1000 mg
*z*_28_	Dacarbazin	151.875	13.98	Vail	158	500 mg
*z*_29_	Pazopanib	332.75	15.68	Tab	913	400 mg
*z*_30_	Irenotican	45	16.92	Vail	110	40 mg
*z*_31_	Ca-folinat	45	2.21	Vial	123	50 mg
*z*_32_	Mesna	39	1.23	Vial	786	200 mg
*z*_33_	Vincristine -2-	34.375	1.1	Vial	332	1 mg
*z*_34_	Etopside	112	2	Vail	170	100 mg
*z*_35_	Bleomycin	45	11.78	Vial	240	15 mg
*z*_36_	Vinblastin -1-	58.5	5.7	Vial	286	10 mg
*z*_37_	Filgrastim 30U.i	116	10.34	Inj	2108	10 mg
*z*_38_	Fludarabine	126	68	Vial	41	50 mg
*z*_39_	Zoladex	495	420	Inj	52	10.8 mg
*z*_40_	Liposomol Doxorubcin	210	137.53	Vial	168	20 mg

The article "Healthcare's Sustainable Resource Planning Using Neutrosophic Goal Programming" was published in 2022. Journal: J Healthc Eng.

**Table 5:** The obtained budgets using GP model.

Year		2018	2020	2024	2028	2032	2036	2040	2044	2048	GR (%)
TB	Cost	316705.7	426305.1	585093.9	920536.3	1263664	1586187	1921383	2258103	2580579	13
TBS	Cost	87600	157440	259200	494640	720480	943200	1178640	1401120	1623840	6
	(%)	28	37	44	54	57	59	61	62	63	
TBM	Cost	26000	32800	57400	92200	144800	179400	214200	263600	298200	9
	(%)	8	8	10	10	11	11	11	12	12	
TBD	Cost	203105.7	236065.1	268493.9	333696.3	398384.2	463587.2	528543.1	593383	658539.2	32
	(%)	64	55	46	36	32	29	28	26	26	

**Table 6:** The number and corresponding cost of staff obtained using GP model.

Staff		*x*_1_	*x*_2_	*x*_3_	*x*_4_	*x*_5_	*x*_6_	*x*_7_	*x*_8_	Total
		Oncologists	General doctors	Radiologists	Pharmacists	Lab technician	X-ray technician	Nurses	Other staff	
2018	No.	2	2	3	2	3	2	4	3	21
	Ratio (%)	10	10	14	10	14	10	19	14	100
	Cost	19200	7680	17280	6720	10080	6240	9600	10800	87600
2020	No.	4	3	5	1	5	3	13	5	39
	Ratio (%)	10	8	13	3	13	8	33	13	100
	Cost	38400	11520	28800	3360	16800	9360	31200	18000	157440
2024	No.	6	5	9	1	9	3	23	9	65
	Ratio (%)	9	8	14	2	14	5	35	14	100
	Cost	57600	19200	51840	3360	30240	9360	55200	32400	259200
2028	No.	12	9	17	2	17	6	43	17	123
	Ratio (%)	10	7	14	2	14	5	35	14	100
	Cost	115200	34560	97920	6720	57120	18720	103200	61200	494640
2032	No.	17	13	25	3	25	9	63	25	180
	Ratio (%)	9	7	14	2	14	5	35	14	100
	Cost	163200	49920	144000	10080	84000	28080	151200	90000	720480
2036	No.	22	17	33	4	33	11	83	33	236
	Ratio (%)	9	7	14	2	14	5	35	14	100
	Cost	211200	65280	190080	13440	110880	34320	199200	118800	943200
2040	No.	28	21	41	5	41	14	103	41	294
	Ratio (%)	10	7	14	2	14	5	35	14	100
	Cost	268800	80640	236160	16800	137760	43680	247200	147600	1178640
2044	No.	33	25	49	5	49	17	123	49	350
	Ratio (%)	9	7	14	1	14	5	35	14	100
	Cost	316800	96000	282240	16800	164640	53040	295200	176400	1401120
2048	No.	38	29	57	6	57	19	143	57	406
	Ratio (%)	9	7	14	1	14	5	35	14	100
	Cost	364800	111360	328320	20160	191520	59280	343200	205200	1623840
GR (%)	6	8	6	35	6	11	3	6	6	

The article "Healthcare's Sustainable Resource Planning Using Neutrosophic Goal Programming" was published in 2022. Journal: J Healthc Eng.

**Table 7:** The number with the corresponding cost of medical devices obtained using GP model.

Medical devices		*y*_1_	*y*_2_	*y*_3_	*y*_4_	*y*_5_	*y*_6_	*y*_7_	Total
		Blood test	Chemistry apparatus	Oncology indications	Ultrasonic	X-ray	Mammogram	Other devices	
2018	No.	1	1	1	1	1	1	4	10
	Ratio (%)	10	10	10	10	10	10	40	100
	Cost	4200	4800	6660	3200	3200	3200	800	26060
2020	No.	2	1	1	1	1	1	17	24
	Ratio (%)	8	4	4	4	4	4	71	100
	Cost	8400	4800	6660	3200	3200	3200	3400	32860
2024	No.	3	2	2	2	2	1	30	42
	Ratio (%)	7	5	5	5	5	2	71	100
	Cost	12600	9600	13320	6400	6400	3200	6000	57520
2028	No.	5	3	3	3	3	2	57	76
	Ratio (%)	7	4	4	4	4	3	75	100
	Cost	21000	14400	19980	9600	9600	6400	11400	92380
2032	No.	7	5	5	5	5	3	84	114
	Ratio (%)	6	4	4	4	4	3	74	100
	Cost	29400	24000	33300	16000	16000	9600	16800	145100
2036	No.	9	6	6	6	6	4	110	147
	Ratio (%)	6	4	4	4	4	3	75	100
	Cost	37800	28800	39960	19200	19200	12800	22000	179760
2040	No.	11	7	7	7	7	5	137	181
	Ratio (%)	6	4	4	4	4	3	76	100
	Cost	46200	33600	46620	22400	22400	16000	27400	214620
2044	No.	13	9	9	9	9	5	164	218
	Ratio (%)	6	4	4	4	4	2	75	100
	Cost	54600	43200	59940	28800	28800	16000	32800	264140
2048	No.	15	10	10	10	10	6	190	251
	Ratio (%)	6	4	4	4	4	2	76	100
	Cost	63000	48000	66600	32000	32000	19200	38000	298800
GR (%)	7	11	11	11	11	18	2	4	

**Table 8:** The quantities of medical drugs obtained using the GP model.

Medical drug names	2018	2020	2024	2028	2032	2036	2040	2044	2048	GR (%)
*z*_1_	13503	15664	17824	22145	26466	30787	35108	39429	43750	32
*z*_2_	80	93	106	132	157	183	208	234	260	32
*z*_3_	484	562	639	794	949	1104	1259	1414	1569	32
*z*_4_	1061	1231	1401	1741	2080	2420	2759	3099	3438	32
*z*_5_	1049	1217	1385	1721	2057	2392	2728	3064	3399	32
*z*_6_	366	425	484	601	718	835	952	1069	1186	32
*z*_7_	610	708	806	1001	1196	1391	1586	1782	1977	32
*z*_8_	694	806	917	1139	1361	1583	1805	2027	2249	32
*z*_9_	155	180	205	255	304	354	403	453	503	32
*z*_10_	605	702	799	993	1186	1380	1573	1767	1961	32
*z*_11_	4535	5261	5987	7438	8889	10340	11791	13243	14694	32
*z*_12_	210	244	278	345	412	479	546	614	681	32
*z*_13_	275	319	363	451	539	627	715	803	891	32
*z*_14_	155	180	205	255	304	354	403	453	503	32
*z*_15_	110	128	146	181	216	251	286	322	357	32
*z*_16_	226	263	299	371	443	516	588	660	733	32
*z*_17_	6374	7394	8414	10454	12494	14533	16573	18613	20652	32
*z*_18_	778	903	1027	1276	1525	1774	2023	2272	2521	32
*z*_19_	790	917	1043	1296	1549	1802	2054	2307	2560	32
*z*_20_	756	877	998	1240	1482	1724	1966	2208	2450	32
*z*_21_	152	177	201	250	298	347	396	444	493	32
*z*_22_	213	248	282	350	418	486	554	622	691	32
*z*_23_	2575	2987	3399	4223	5047	5871	6695	7519	8343	32
*z*_24_	2002	2323	2643	3284	3924	4565	5206	5846	6487	32
*z*_25_	281	326	371	461	551	641	731	821	911	32
*z*_26_	262	304	346	430	514	598	682	766	849	32
*z*_27_	411	477	543	675	806	938	1069	1201	1332	32
*z*_28_	158	184	209	260	310	361	411	462	512	32
*z*_29_	913	1060	1206	1498	1790	2082	2374	2666	2959	32
*z*_30_	110	128	146	181	216	251	286	322	357	32
*z*_31_	123	143	163	202	242	281	320	360	399	32
*z*_32_	786	912	1038	1290	1541	1793	2044	2296	2547	32
*z*_33_	332	386	439	545	651	757	864	970	1076	32
*z*_34_	170	198	225	279	334	388	442	497	551	32
*z*_35_	240	279	317	394	471	548	624	701	778	32
*z*_36_	286	332	378	470	561	653	744	836	927	32
*z*_37_	2108	2446	2783	3458	4132	4807	5481	6156	6830	32
*z*_38_	41	48	55	68	81	94	107	120	133	32
*z*_39_	52	61	69	86	102	119	136	152	169	32
*z*_40_	168	195	222	276	330	384	437	491	545	32
Sum	44199	51288	58361	72509	86646	100793	114929	129081	143223	32

The article "Healthcare's Sustainable Resource Planning Using Neutrosophic Goal Programming" was published in 2022. Journal: J Healthc Eng.

**Table 9:** The negative deviational variables obtained using GP model.

Negative deviations	2018	2020	2024	2028	2032	2036	2040	2044	2048
N1	48000	0	0	0	0	0	0	0	0
N2	0	0	0	0	0	0	0	0	0
N3	0	0	0.2	0	0	0	0	0	0
N4	48000	0	0	0	0	0	0	0	0

**Table 10:** The positive deviational variables obtained using the GP model.

Positive deviations	2018	2020	2024	2028	2032	2036	2040	2044	2048
P1	0	288	160415.8	562485.6	965498.4	1344271	1755267	2148461	2527308
P2	0	144	80208	272256	454704	634032	826080	1005168	1184496
P3	0	0	0	17973.6	56090.4	76207.2	103107.3	138125.4	158316.4
P4	0	144	80208	272256	454704	634032	826080	1005168	1184496
PX1	1.333333	0.666667	0	0.666667	0.333333	0	0.666667	0.333333	0
PX2	1.5	0.5	0.5	0.5	0.5	0.5	0.5	0.5	0.5
PX3	2	0	0	0	0	0	0	0	0
PX4	1.9	0.5	0.1	0.3	0.5	0.7	0.9	0.1	0.3
PX5	2	0	0	0	0	0	0	0	0
PX6	1.666667	1.333333	0	0.333333	0.666667	0	0.333333	0.666667	0
PX7	1.5	0.5	0.5	0.5	0.5	0.5	0.5	0.5	0.5
PX8	2	0	0	0	0	0	0	0	0
PY1	0.75	0.75	0.75	0.75	0.75	0.75	0.75	0.75	0.75
PY2	0.833333	0.166667	0.5	0.166667	0.833333	0.5	0.166667	0.833333	0.5
PY3	0.833333	0.166667	0.5	0.166667	0.833333	0.5	0.166667	0.833333	0.5
PY4	0.833333	0.166667	0.5	0.166667	0.833333	0.5	0.166667	0.833333	0.5
PY5	0.833333	0.166667	0.5	0.166667	0.833333	0.5	0.166667	0.833333	0.5
PY6	0.9	0.5	0.1	0.3	0.5	0.7	0.9	0.1	0.3
PY7	0.666667	0.333333	0	0.333333	0.666667	0	0.333333	0.666667	0

The article "Healthcare's Sustainable Resource Planning Using Neutrosophic Goal Programming" was published in 2022. Journal: J Healthc Eng.

**Table 11:** Values of the neutrosophic variables.

${\tilde{\tau }}_{a}^{N}$	*a*	(*a*, *l*_*μ*_, *r*_*μ*_; *w*_*a*_), (*a*, *l*_*σ*_, *r*_*σ*_; *u*_*a*_), (*a*, *l*_*ν*_, *r*_*ν*_; *y*_*a*_)	*α*	*β*	*γ*
${\tilde{TB}}^{N}$	570860	(100000,200000; 0.9), (30000,40000; 0.3), (800000,100000; 0.5)	0.1	0.9	0.8
${\left(\tilde{TBS}\right)}^{N}$	135600	(13000,100000; 0.9), (18000,15000; 0.3), (20000,30000; 0.5)	0.1	0.9	0.8
${\left(\tilde{TBM}\right)}^{N}$	45260	(1000,5000; 0.9), (9000,10000; 0.3), (10000,15000; 0.5)	0.1	0.9	0.8
${\left(\tilde{TB\;D}\right)}^{N}$	390000	(10000,100000; 0.9), (20000,30000; 0.3), (15000,20000; 0.5)	0.1	0.9	0.8

**Table 12:** Budgets results of NGP model.

Year		2018	2020	2024	2028	2032	2036	2040	2044	2048	GR (%)
TB	Cost	359415.6	407990.3	672852.8	920536.3	1196277	1579471	1921383	2288403	2613624	15
TBS	Cost	120960	151920	326160	494640	684000	940800	1178640	1425840	1651680	8
	(%)	34	37	48	54	57	60	61	62	63	
TBM	Cost	26600	28000	62000	92200	122000	179200	214200	264000	298600	10
	(%)	7	7	9	10	10	11	11	12	11	
TBD	Cost	211855.6	228070.3	284692.8	333696.3	390277.3	459470.6	528543.1	598563.4	663344	33
	(%)	59	56	42	36	33	29	28	26	25	

**Table 13:** The staff numbers obtained using the NGP model.

Staff		*x*_1_	*x*_2_	*x*_3_	*x*_4_	*x*_5_	*x*_6_	*x*_7_	*x*_8_	Total
		Oncologists	General doctors	Radiologists	Pharmacists	Lab technician	X-ray technician	Nurses	Other staff	
2018	No.	3	3	4	2	4	2	7	4	29
	Ratio (%)	10	10	14	7	14	7	24	14	100
	Cost	28800	11520	23040	6720	13440	6240	16800	14400	120960
2020	No.	4	2	6	1	6	3	10	4	36
	Ratio (%)	11	6	17	3	17	8	28	11	100
	Cost	38400	7680	34560	3360	20160	9360	24000	14400	151920
2024	No.	8	6	11	2	11	4	28	11	81
	Ratio (%)	10	7	14	2	14	5	35	14	100
	Cost	76800	23040	63360	6720	36960	12480	67200	39600	326160
2028	No.	12	9	17	2	17	6	43	17	123
	Ratio (%)	10	7	14	2	14	5	35	14	100
	Cost	115200	34560	97920	6720	57120	18720	103200	61200	494640
2032	No.	16	12	24	3	24	8	60	24	171
	Ratio (%)	9	7	14	2	14	5	35	14	100
	Cost	153600	46080	138240	10080	80640	24960	144000	86400	684000
2036	No.	22	17	33	4	33	11	82	33	235
	Ratio (%)	9	7	14	2	14	5	35	14	100
	Cost	211200	65280	190080	13440	110880	34320	196800	118800	940800
2040	No.	28	21	41	5	41	14	103	41	294
	Ratio (%)	10	7	14	2	14	5	35	14	100
	Cost	268800	80640	236160	16800	137760	43680	247200	147600	1178640
2044	No.	34	25	50	5	50	17	124	50	355
	Ratio (%)	10	7	14	1	14	5	35	14	100
	Cost	326400	96000	288000	16800	168000	53040	297600	180000	1425840
2048	No.	39	29	58	6	58	20	144	58	412
	Ratio (%)	9	7	14	1	14	5	35	14	100
	Cost	374400	111360	334080	20160	194880	62400	345600	208800	1651680
GR (%)	8	11	8	35	8	11	5	8	8	

The article "Healthcare's Sustainable Resource Planning Using Neutrosophic Goal Programming" was published in 2022. Journal: J Healthc Eng.

**Table 14:** The medical devices numbered obtained using NGP model.

Medical devices		*y*_1_	*y*_2_	*y*_3_	*y*_4_	*y*_5_	*y*_6_	*y*_7_	Total
		Blood Test	Chemistry apparatus	Oncology indications	Ultrasonic	X-ray	Mammogram	Other devices	
2018	No.	1	1	1	1	1	1	7	13
	Ratio (%)	8	8	8	8	8	8	54	100
	Cost	4200	4800	6660	3200	3200	3200	1400	26660
2020	No.	1	1	1	1	1	1	14	20
	Ratio (%)	5	5	5	5	5	5	70	100
	Cost	4200	4800	6660	3200	3200	3200	2800	28060
2024	No.	3	2	2	2	2	2	37	50
	Ratio (%)	6	4	4	4	4	4	74	100
	Cost	12600	9600	13320	6400	6400	6400	7400	62120
2028	No.	5	3	3	3	3	2	57	76
	Ratio (%)	7	4	4	4	4	3	75	100
	Cost	21000	14400	19980	9600	9600	6400	11400	92380
2032	No.	6	4	4	4	4	3	80	105
	Ratio (%)	6	4	4	4	4	3	76	100
	Cost	25200	19200	26640	12800	12800	9600	16000	122240
2036	No.	9	6	6	6	6	4	109	146
	Ratio (%)	6	4	4	4	4	3	75	100
	Cost	37800	28800	39960	19200	19200	12800	21800	179560
2040	No.	11	7	7	7	7	5	137	181
	Ratio (%)	6	4	4	4	4	3	76	100
	Cost	46200	33600	46620	22400	22400	16000	27400	214620
2044	No.	13	9	9	9	9	5	166	220
	Ratio (%)	6	4	4	4	4	2	75	100
	Cost	54600	43200	59940	28800	28800	16000	33200	264540
2048	No.	15	10	10	10	10	6	192	253
	Ratio (%)	6	4	4	4	4	2	76	100
	Cost	63000	48000	66600	32000	32000	19200	38400	299200
GR	7	11	11	11	11	18	4	6	

**Table 15:** The medical drugs quantities obtained using NGP model.

Medical drug names	2018	2020	2024	2028	2032	2036	2040	2044	2048	GR (%)
*z*_1_	14044	15124	18905	22145	25926	30517	35108	39753	44074	33
*z*_2_	84	90	112	132	154	181	208	236	262	33
*z*_3_	504	543	678	794	930	1094	1259	1425	1580	33
*z*_4_	1104	1189	1486	1741	2038	2398	2759	3124	3464	33
*z*_5_	1091	1175	1469	1721	2015	2371	2728	3089	3424	33
*z*_6_	381	410	513	601	703	828	952	1078	1195	33
*z*_7_	635	684	854	1001	1172	1379	1586	1796	1992	33
*z*_8_	722	778	972	1139	1333	1569	1805	2044	2266	33
*z*_9_	162	174	217	255	298	351	403	457	506	33
*z*_10_	630	678	847	993	1162	1368	1573	1782	1975	33
*z*_11_	4717	5080	6349	7438	8708	10250	11791	13352	14803	33
*z*_12_	219	236	294	345	404	475	546	619	686	33
*z*_13_	286	308	385	451	528	622	715	810	898	33
*z*_14_	162	174	217	255	298	351	403	457	506	33
*z*_15_	115	124	154	181	212	249	286	324	360	33
*z*_16_	236	254	317	371	434	511	588	666	738	33
*z*_17_	6629	7139	8924	10454	12239	14406	16573	18766	20805	33
*z*_18_	810	872	1090	1276	1494	1759	2023	2291	2540	33
*z*_19_	822	885	1106	1296	1517	1786	2054	2326	2579	33
*z*_20_	787	847	1059	1240	1452	1709	1966	2226	2468	33
*z*_21_	159	171	213	250	292	344	396	448	497	33
*z*_22_	222	239	299	350	409	482	554	628	696	33
*z*_23_	2678	2884	3605	4223	4944	5820	6695	7581	8405	33
*z*_24_	2083	2243	2803	3284	3844	4525	5206	5894	6535	33
*z*_25_	293	315	394	461	540	636	731	828	918	33
*z*_26_	273	294	367	430	504	593	682	772	856	33
*z*_27_	428	461	576	675	790	929	1069	1210	1342	33
*z*_28_	165	177	222	260	304	358	411	466	516	33
*z*_29_	950	1023	1279	1498	1753	2064	2374	2688	2981	33
*z*_30_	115	124	154	181	212	249	286	324	360	33
*z*_31_	128	138	173	202	237	278	320	363	402	33
*z*_32_	818	881	1101	1290	1510	1777	2044	2314	2566	33
*z*_33_	346	372	465	545	638	751	864	978	1084	33
*z*_34_	177	191	238	279	327	385	442	501	555	33
*z*_35_	250	269	336	394	461	543	624	707	784	33
*z*_36_	298	321	401	470	550	647	744	842	934	33
*z*_37_	2193	2361	2952	3458	4048	4765	5481	6206	6881	33
*z*_38_	43	46	58	68	79	93	107	121	134	33
*z*_39_	55	59	73	86	100	118	136	154	170	34
*z*_40_	175	189	236	276	323	380	437	495	549	33
Sum	45989	49522	61893	72509	84882	99911	114929	130141	144286	33

The article "Healthcare's Sustainable Resource Planning Using Neutrosophic Goal Programming" was published in 2022. Journal: J Healthc Eng.

**Table 16:** The negative deviational variables obtained using the NGP model.

Negative deviations	2018	2020	2024	2028	2032	2036	2040	2044	2048
N1	0	0	0	0	0	0	0	0	0
N2	0	0	0	0	0	0	0	0	0
N3	20064	0	0	0	0	0	0	0	0
N4	0	0	0	0	0	0	0	0	0

**Table 17:** The positive deviational variables obtained using the NGP model.

Positive deviations	2018	2020	2024	2028	2032	2036	2040	2044	2048
P1	0	96	276448.6	691594.3	888565.6	1352026	1960156	2190713	2575798
P2	20064	48	136320	249634.3	423648	634344	790216.4	1026634	1209082
P3	0	0	3808.571	15674.12	41269.57	83338.05	99665.71	137445.5	157635
P4	0	48	136320	249634.3	423648	634344	790216.4	1026634	1209082
PX1	1.666667	1.333333	0.666667	0.666667	0	0.333333	0.666667	0.933333	0.6
PX2	2	0	0.5	0.5	0	0.75	0.5	0.2	0.2
PX3	2	2	0	0	0	0.5	0	0.4	0.4
PX4	1.8	0.6	0.9	0.3	0.6	0.75	0.9	4.00E-02	0.24
PX5	2	2	0	0	0	0.5	0	0.4	0.4
PX6	1.333333	1.666667	0.333333	0.333333	0	0.166667	0.333333	0.466667	0.8
PX7	2	0	0.5	0.5	0	0.75	0.5	0	0
PX8	2	0	0	0	0	0.5	0	0.4	0.4
PY1	0.5	0	0.25	0.75	0	0.875	0.75	0.6	0.6
PY2	0.666667	0.333333	0.166667	0.166667	0	0.583333	0.166667	0.733333	0.4
PY3	0.666667	0.333333	0.166667	0.166667	0	0.583333	0.166667	0.733333	0.4
PY4	0.666667	0.333333	0.166667	0.166667	0	0.583333	0.166667	0.733333	0.4
PY5	0.666667	0.333333	0.166667	0.166667	0	0.583333	0.166667	0.733333	0.4
PY6	0.8	0.6	0.9	0.3	0.6	0.75	0.9	4.00E-02	0.24
PY7	0.333333	0.666667	0.333333	0.333333	0	0.666667	0.333333	0.666667	0

**Table 18:** Values of the neutrosophic variables.

${\tilde{\tau }}_{g}^{N}$	*g*	〈 *g*_1_, *g*_2_, *g*_3_〉
${\tilde{\text{TB}}}^{N}$	570860	〈 615304.4, 575145.7143, 590860〉
${\left(\tilde{\text{TBS}}\right)}^{N}$	135600	〈 174266.7, 134314.3, 131600〉
${\left(\tilde{\text{TBM}}\right)}^{N}$	45260	〈 47037.78, 45688.57, 47260〉
${\left(\tilde{\text{TBD}}\right)}^{N}$	390000	〈 430000, 394285.7, 392000〉

**Table 19:** The obtained budgets using NMCGP model.

Year		2018	2020	2024	2028	2032	2036	2040	2044	2048	GR (%)
TB	Cost	337882.6	512647.8	585093.9	874117.3	1299211	1586187	1940197	2164600	2618038	14
TBS	Cost	90720	208320	259200	461280	747600	943200	1193760	1347120	1654080	6
	(%)	15	36	32	50	57	59	61	62	63	
TBM	Cost	27200	52000	57400	87400	145400	179400	214400	240200	298800	10
	(%)	10	8	7	9	11	11	11	12	12	
TBD	Cost	219962.6	252327.8	268493.9	325437.3	406211.4	463587.2	532037.4	577280.5	665157.6	34
	(%)	76	56	61	41	32	29	28	26	26	

The article "Healthcare's Sustainable Resource Planning Using Neutrosophic Goal Programming" was published in 2022. Journal: J Healthc Eng.

**Table 20:** The staff number obtained using the NMCGP model.

Staff		*x*_1_	*x*_2_	*x*_3_	*x*_4_	*x*_5_	*x*_6_	*x*_7_	*x*_8_
		Oncologists	General doctors	Radiologists	Pharmacists	Lab technician	X-ray technician	Nurses	Other staff	Total
2018	No.	2	2	3	1	3	1	8	3	23
	Ratio (%)	9	9	13	4	13	4	35	13	100
	Cost	19200	7680	17280	3360	10080	3120	19200	10800	90720
2020	No.	5	4	7	1	7	3	18	7	52
	Ratio (%)	10	8	13	2	13	6	35	13	100
	Cost	48000	15360	40320	3360	23520	9360	43200	25200	208320
2024	No.	6	5	9	1	9	3	23	9	65
	Ratio (%)	9	8	14	2	14	5	35	14	100
	Cost	57600	19200	51840	3360	30240	9360	55200	32400	259200
2028	No.	11	8	16	2	16	6	40	16	115
	Ratio (%)	10	7	14	2	14	5	35	14	100
	Cost	105600	30720	92160	6720	53760	18720	96000	57600	461280
2032	No.	18	13	26	3	26	9	65	26	186
	Ratio (%)	10	7	14	2	14	5	35	14	100
	Cost	172800	49920	149760	10080	87360	28080	156000	93600	747600
2036	No.	22	17	33	4	33	11	83	33	236
	Ratio (%)	9	7	14	2	14	5	35	14	100
	Cost	211200	65280	190080	13440	110880	34320	199200	118800	943200
2040	No.	28	21	42	5	42	14	104	42	298
	Ratio (%)	9	7	14	2	14	5	35	14	100
	Cost	268800	80640	241920	16800	141120	43680	249600	151200	1193760
2044	No.	32	24	47	5	47	16	118	47	336
	Ratio (%)	10	7	14	1	14	5	35	14	100
	Cost	307200	92160	270720	16800	157920	49920	283200	169200	1347120
2048	No.	39	29	58	6	58	20	145	58	413
	Ratio (%)	9	7	14	1	14	5	35	14	100
	Cost	374400	111360	334080	20160	194880	62400	348000	208800	1654080
GR (%)	6	8	6	18	6	6	6	6	6	

**Table 21:** The medical devices numbered obtained using NMCGP model.

Medical devices		*y*_1_	*y*_2_	*y*_3_	*y*_4_	*y*_5_	*y*_6_	*y*_7_	Total
		Blood test	Chemistry apparatus	Oncology indications	Ultrasonic	X-ray	Mammogram	Other devices	
2018	No.	1	1	1	1	1	1	10	16
	Ratio (%)	6	6	6	6	6	6	63	100
	Cost	4200	4800	6660	3200	3200	3200	2000	27260
2020	No.	2	2	2	2	2	1	24	35
	Ratio (%)	6	6	6	6	6	3	69	100
	Cost	8400	9600	13320	6400	6400	3200	4800	52120
2024	No.	3	2	2	2	2	1	30	42
	Ratio (%)	7	5	5	5	5	2	71	100
	Cost	12600	9600	13320	6400	6400	3200	6000	57520
2028	No.	4	3	3	3	3	2	54	72
	Ratio (%)	6	4	4	4	4	3	75	100
	Cost	16800	14400	19980	9600	9600	6400	10800	87580
2032	No.	7	5	5	5	5	3	87	117
	Ratio (%)	6%	4%	4%	4%	4%	3%	74%	100%
	Cost	29400	24000	33300	16000	16000	9600	17400	145700
2036	No.	9	6	6	6	6	4	110	147
	Ratio (%)	6	4	4	4	4	3	75	100
	Cost	37800	28800	39960	19200	19200	12800	22000	179760
2040	No.	11	7	7	7	7	5	138	182
	Ratio (%)	6	4	4	4	4	3	76	100
	Cost	46200	33600	46620	22400	22400	16000	27600	214820
2044	No.	12	8	8	8	8	5	157	206
	Ratio (%)	6	4	4	4	4	2	76	100
	Cost	50400	38400	53280	25600	25600	16000	31400	240680
2048	No.	15	10	10	10	10	6	193	254
	Ratio (%)	6%	4%	4%	4%	4%	2%	76%	100%
	Cost	63000	48000	66600	32000	32000	19200	38600	299400
GR (%)	7	11	11	11	11	18	6	7	

The article "Healthcare's Sustainable Resource Planning Using Neutrosophic Goal Programming" was published in 2022. Journal: J Healthc Eng.

**Table 22:** Medical drugs quantities obtained using the NMCGP model.

Medicament name	2018	2020	2024	2028	2032	2036	2040	2044	2048	GR (%)
*z*_1_	14584	16744	17824	21605	27006	30787	35324	38349	44182	34
*z*_2_	87	100	106	128	160	183	210	228	262	34
*z*_3_	523	601	639	775	968	1104	1267	1375	1584	34
*z*_4_	1146	1316	1401	1698	2122	2420	2776	3014	3472	34
*z*_5_	1133	1301	1385	1679	2098	2392	2745	2980	3433	34
*z*_6_	396	454	484	586	732	835	958	1040	1198	34
*z*_7_	659	757	806	976	1220	1391	1596	1733	1996	34
*z*_8_	750	861	917	1111	1388	1583	1816	1971	2271	34
*z*_9_	168	193	205	248	310	354	406	441	508	34
*z*_10_	654	751	799	968	1210	1380	1583	1719	1980	34
*z*_11_	4898	5624	5987	7256	9070	10340	11864	12880	14839	34
*z*_12_	227	261	278	336	420	479	550	597	688	34
*z*_13_	297	341	363	440	550	627	720	781	900	34
*z*_14_	168	193	205	248	310	354	406	441	508	34
*z*_15_	119	137	146	176	220	251	288	313	360	34
*z*_16_	245	281	299	362	452	516	592	642	740	34
*z*_17_	6884	7904	8414	10199	12748	14533	16675	18103	20856	34
*z*_18_	841	965	1027	1245	1556	1774	2036	2210	2546	34
*z*_19_	854	980	1043	1264	1580	1802	2067	2244	2585	34
*z*_20_	817	938	998	1210	1512	1724	1978	2148	2474	34
*z*_21_	165	189	201	244	304	347	398	432	498	34
*z*_22_	231	265	282	341	426	486	558	605	697	34
*z*_23_	2781	3193	3399	4120	5150	5871	6737	7313	8426	34
*z*_24_	2163	2483	2643	3204	4004	4565	5238	5686	6551	34
*z*_25_	304	349	371	450	562	641	736	799	920	34
*z*_26_	283	325	346	420	524	598	686	745	858	34
*z*_27_	444	510	543	658	822	938	1076	1168	1345	34
*z*_28_	171	196	209	253	316	361	414	449	517	34
*z*_29_	987	1133	1206	1461	1826	2082	2389	2593	2988	34
*z*_30_	119	137	146	176	220	251	288	313	360	34
*z*_31_	133	153	163	197	246	281	322	350	403	34
*z*_32_	849	975	1038	1258	1572	1793	2057	2233	2572	34
*z*_33_	359	412	439	532	664	757	869	943	1087	34
*z*_34_	184	211	225	272	340	388	445	483	557	34
*z*_35_	260	298	317	384	480	548	628	682	786	34
*z*_36_	309	355	378	458	572	653	749	813	936	34
*z*_37_	2277	2614	2783	3373	4216	4807	5515	5987	6898	34
*z*_38_	45	51	55	66	82	94	108	117	135	35
*z*_39_	57	65	69	84	104	119	137	148	171	35
*z*_40_	182	209	222	269	336	384	440	478	550	34
Sum	47753	54825	58361	70730	88398	100793	115647	125546	144637	34

The article "Healthcare's Sustainable Resource Planning Using Neutrosophic Goal Programming" was published in 2022. Journal: J Healthc Eng.

**Table 23:** Summary of the comparison between the proposed models.

		2018	2020	2024	2028	2032	2036	2040	2044	2048	GR (%)
Total Budget	GP	316705.7	426305.1	585093.9	920536.3	1263664	1586187	1921383	2258103	2580579	13
	NGP	359415.6	407990.3	672852.8	920536.3	1196277	1579471	1921383	2288403	2613624	15
	MCNGP	337882.6	512647.8	585093.9	874117.3	1299211	1586187	1940197	2164600	2618038	14
Total Staff	GP	21	39	65	123	180	236	294	350	406	6
	NGP	29	36	81	123	171	235	294	355	412	8
	MCNGP	23	52	65	115	186	236	298	336	413	6
Total Devices	GP	10	24	42	76	114	147	181	218	251	4
	NGP	13	20	50	76	105	146	181	220	253	6
	MCNGP	16	35	42	72	117	147	182	206	254	7
Total Medicines	GP	44199	51288	58361	72509	86646	100793	114929	129081	143223	32
	NGP	45989	49522	61893	72509	84882	99911	114929	130141	144286	32
	MCNGP	47753	54825	58361	70730	88398	100793	115647	125546	144637	32
Objective Function	GP	96019.55	581.75	320836	1124976	1931005	2688548	3510540	4296930	5054621	2
	NGP	40147.1	202.2	552902.2	1206541	1777132	2704061	3640260	4381432	5151602	1
	MCNGP	4.65	6.85	29499.45	200538.3	525486.9	808013.9	1166643	1382879	1840569	0

## Data Availability

The data used to support the findings of this study are included within the article.
